This article has been retracted.

# Correlation between Glycated Haemoglobin Level, Cardiac Function, and Prognosis in Patients with Diabetes Mellitus Combined with Myocardial Infarction

**DOI:** 10.1155/2022/2191294

**Published:** 2022-09-23

**Authors:** Guangwei Zeng, Huixian An, Wei Li, Dong Fang, Mengna Sun, Qiangsun Zheng

**Affiliations:** ^1^Department of Cardiology, The Second Affiliated Hospital of Xi'an Jiaotong University, No.157 Xiwu Rd., Xi'an City, Shaanxi 710004, China; ^2^Department of Cardiology, Section 2, Xi'an International Medical Center Hospital, Xi'an City, Shaanxi 710100, China

## Abstract

**Objective:**

This study was to investigate the correlation between glycated haemoglobin (HbA1c) level, cardiac function, and prognosis in patients with diabetes mellitus combined with myocardial infarction.

**Methods:**

Ninety-three patients with type 2 diabetes mellitus combined with acute myocardial infarction who were hospitalized and treated in our hospital from January 2021 to June 2021 were recruited for prospective analysis and equally divided into group A (HbA1c < 6.5%), group B (6.5% ≤ HbA1c ≤ 8.5%), and group C (HbA1c > 8.5%) using the random number table method, with 31 patients in each group. General data of patients were collected on admission and blood glucose and cardiac function indexes were measured; the incidence of myocardial infarction and death during the follow-up period was recorded at 6 months after discharge.

**Results:**

There was a significant difference in blood glucose (FBG) and HbA1c levels at fasting between the three groups (*P* < 0.05). There were statistically significant differences in plasma levels of N-terminal probrain natriuretic peptide (NT-proBNP) and uric acid (UA), left ventricular end diastolic diameter (LVEDD), left ventricular end systolic volume (LVESV), left ventricular ejection fraction (LVEF), and cardiac function classification of the New York Heart Association (NYHA) among the three groups (*P* < 0.05). By statistical analysis, the HbA1c level was positively correlated with FBG, NT-proBNP, UA, LVEDD, LVESD, and NYHA grades but negatively correlated with LVEF (*P* < 0.05). The incidence rate of myocardial infarction and mortality was significantly higher in group C than in groups A and B (*P* < 0.05).

**Conclusion:**

HbA1c level in patients with diabetes mellitus combined with myocardial infarction is closely related to the degree of cardiac function damage. Glycated haemoglobin levels are associated with the development of cardiac insufficiency in patients with acute myocardial infarction; glycated haemoglobin is also an independent predictor of major adverse cardiovascular events. Reasonable and effective blood glucose control is of great significance to the prognosis of patients.

## 1. Introduction

Acute myocardial infarction is a common cardiovascular disease that could be life-threatening and significantly reduce the quality of life of patients. According to some literatures, the amount of people suffering from cardiovascular diseases in China reaches approximately 230 million, and there is epidemiological data indicating that one cardiovascular disease death occurs every 12 seconds in China. Acute heart attacks are common and prevalent in emergency departments, with rapid onset and progression, and could be fatal if not treated promptly and effectively [1]. The prognosis does not remain optimistic, with an in-hospital mortality rate of approaching 30% [2]. Studies have established that approximately 16.7% of patients with acute myocardial infarction have diabetes [3], and the combination of acute myocardial infarction and diabetes mellitus significantly increases the clinical mortality in patients [4]. An additional study has illustrated that disturbances in glucose metabolism due to fluctuations in blood glucose fluctuation are one of the leading factors in the mortality of patients with acute myocardial infarction [5]. Early diagnosis of diabetes and effective control of blood glucose in the patient's body could effectively improve the prognosis of the disease and minimize the damage caused by diabetes. Diabetes is a common underlying metabolic disease with many complications and requires lifelong medication to control blood glucose levels. Studies have previously documented that the development of complications from diabetes mellitus affects glycaemic control and is a major cause of mortality in patients. There is a strong association between abnormal glucose metabolism and the development and clinical prognosis of coronary heart disease, in which has been reported that a 1% increase in glycosylated haemoglobin levels is associated with a 20% increase in the incidence of adverse cardiac events [6, 7].

Glycated haemoglobin (HbA1c) is an essential criterion for evaluating long-term blood glucose control in clinical practice [8]. HbA1c is the product of a nonenzymatic reaction in which glucose in the blood is bound to haemoglobin in the form red blood cells. The hyperglycaemic state plays a major role in the activation of oxidative stress and leads to a massive production of mitochondrial peroxides, triggering multiple metabolic pathways of glucose-mediated vascular damage. Glucose could react with various proteins to form glycosylated end products, thereby promoting long-term complications such as diabetes, plaque formation, and atherosclerosis [9]. These effects accumulate gradually during prolonged exposure to high blood glucose levels. A prolonged hyperglycaemic state accelerates the normal physiological process of glucose binding to haemoglobin to form HbA1c, resulting in reduced synthesis of 2,3-diphosphoglycerol and increased affinity of haemoglobin for oxygen that is not readily dissociated, thereby exacerbating myocardial ischaemia and hypoxia [10].

In this study, 93 patients with type 2 diabetes mellitus combined with acute myocardial infarction admitted to our hospital from January 2021 to June 2021 were equally enrolled and divided into group A (HbA1c < 6.5%), group B (6.5% ≤ HbA1c ≤ 8.5%), and group C (HbA1c > 8.5%), reflecting the different levels of blood glucose control of the patients. A prospective analysis was conducted on the incidence of recurrent myocardial infarction and death and the correlation between HbA1c level with cardiac function and prognosis. The results are reported as follows.

## 2. Materials and Methods

### 2.1. General Data

A total of 93 patients with type 2 diabetes mellitus combined with acute myocardial infarction who were hospitalized and treated in our hospital from January 2021 to June 2021 were recruited for prospective analysis and equally divided into group A (HbA1c < 6.5%), group B (6.5% ≤ HbA1c ≤ 8.5%), and group C (HbA1c > 8.5%) using the random number table method, with 31 patients in each group.

With a sample size of 31 subjects observed with A, B, and C, the trial will have more than 90% power to detect a difference between A, B, and C in the proportion of subjects with a myocardial infarction and death greater than 10%, given that the probabilities to achieve this myocardial infarction and death are 10% for A and 14% for B.

The trial was conducted according to Good Clinical Practice guidelines developed by the International Council for Harmonisation and in compliance with the trial protocol. The protocol was approved by the institutional review boards or independent ethics committees at each site (Approval No. NU-YU20210102). All patients provided written informed consent per Declaration of Helsinki principles. An independent data monitoring committee monitored safety and efficacy data.

### 2.2. Inclusion and Exclusion Criteria

#### 2.2.1. Inclusion Criteria

1. Patients aged 18-80 years
2. Patients meeting the diagnostic criteria of type 2 diabetes [11]
3. Patients with a diagnosis of ST-segment elevation myocardial infarction [12] and *onset* *time* < 12 *h*
4. Patients who have been on regular hypoglycaemic therapy for more than 6 months
5. Patients with typical chest pain symptoms lasting more than 30 minutes and ST-segment elevation in two adjacent *leads* ≥ 2 *mm* or within 18 hours of onset, with evidence of ongoing ischaemia or haemodynamic instability

#### 2.2.2. Exclusion Criteria

1. Patients with serious infectious diseases or autoimmune diseases and trauma
2. Patients with malignant tumors
3. Patients with diabetic complications, such as diabetic foot and diabetic ketoacidosis
4. Patients with old myocardial infarction or coronary artery caused by various reasons and angiography failure
5. Patients with acute liver and kidney insufficiency
6. Pregnant or lactating women

### 2.3. Methods

#### 2.3.1. Data Collection

General information of patients such as age, gender, height, weight, hypertension, hyperlipidemia, history of cardiovascular disease, hypoglycaemic therapy, and infarction site was collected at enrollment.

(1) $$\begin{array}{c} \text{Body mass index }\left(\text{BMI}\right)={\left[\frac{\text{weight }\left(\text{kg}\right)}{\text{height }\left(\text{m}\right)}\right]}^{2}. \end{array}$$

#### 2.3.2. Blood Glucose Indicators

Patients had their venous blood drawn during fasting and centrifuged at 3000 r/min for 20 min; then, the HbA1c level was determined by cationic high-performance liquid chromatography. The kit was purchased from Shanghai Yudole Biotechnology Co., Ltd. Fasting blood-glucose (FBG) levels were determined by enzyme-linked immunosorbent assay. The kit was purchased from Shanghai Jichun Industrial Co., Ltd. (Cat. No. JCSW2609).

#### 2.3.3. Cardiac Function Indicators

Fasting venous blood was drawn from patients and centrifuged at 3000 r/min for 20 min to separate the serum, then plasma, and the level of N-terminal probrain natriuretic peptide (NT-proBNP) in the plasma was determined by enzyme-linked immunosorbent assay. The kit was purchased from Wuhan Fein Biotechnology Co., Ltd. (Cat. No. EH0350), and an automatic biochemical analyser (Shenzhen Mindray, BS-280) was used to measure serum uric acid (UA) levels. The left ventricular end diastolic diameter (LVEDD), left ventricular end systolic volume (LVESV), and left ventricular ejection fraction (LVEF) were measured by echocardiography. The cardiac cycle was averaged, and the instrument used the cardiovascular ultrasound diagnostic apparatus (iE33 type) produced by Philips. The New York Heart Association (NYHA) was used to evaluate the cardiac function of patients.

*Grade I*: the patient's general activities were basically unrestricted. *Grade II*: patients were asymptomatic at rest, but physical activity was slightly restricted. *Grade III*: the patient's physical activity was markedly restricted, and activity less than normal could cause symptoms of palpitations, dyspnea, and angina pectoris. *Grade IV*: patients had inability to perform any physical activity, and the above symptoms could occur at rest.

#### 2.3.4. Prognosis

The patients were followed up monthly by outpatient and telephone for 6 months after discharge, and the occurrence of myocardial infarction and death was recorded during the follow-up period.

### 2.4. Statistical Analysis

If the parameter beta is either a difference of means, a log odds ratio, or a log hazard ratio, then it is reasonable to assume that *b* is unbiased and normally distributed.

SPSS 20.0 software was used for statistical analysis of the data. The measurement data conformed to a normal distribution and were expressed as $\left(\bar{x}\pm s\right)$, and the three groups were compared using one-way analysis of one-way ANOVA and Snk-*q* test for pairwise comparison. The enumeration data were expressed as [*n*(%)], the total number of cases was ≥40, the minimum theoretical frequency > 5, and the chi-square uncorrected method was used. Bivariate correlations conforming to a normal distribution were analysed using Pearson analysis, and those not conforming to a normal distribution were analysed using Spearman's rank correlation. *P* < 0.05 indicated that the difference is statistically significant.

## 3. Results

### 3.1. Comparison of Three Groups of General Data

There were no significant differences between the three groups in terms of age, BMI, length of diabetes, smoking history, hypertension, hyperlipidemia, history of cardiovascular disease, hypoglycaemic medication, and infarct site (*P* > 0.05) (Table 1).

### 3.2. Comparison of Blood Glucose Indicators among the Three Groups

There were significant differences in FBG and HbA1c levels between the three groups of patients (*P* < 0.05) (Table 2).

### 3.3. Comparison of Cardiac Function among the Three Groups

There were substantial variations in the three groups' NT-proBNP and UA levels, as well as LVEDD, LVESV, LVEF, and NYHA grades (*P* < 0.05) (Table 3).

### 3.4. Correlation Analysis between HbA1c and Various Indicators

There was a significant positive correlation between patients' HbA1c levels and FBG, NT-proBNP, UA, LVEDD, LVESD, and NYHA grades, while a significantly negative correlation with LVEF (*P* < 0.05) (Table 4).

### 3.5. Comparison of Prognosis among the Three Groups

The incidence of recurrence rate and mortality of patients in group C was significantly higher than those in groups A and B (*P* < 0.05) (Table 5).

## 4. Discussion

Acute myocardial infarction is typically divided into ST-segment elevation myocardial infarction and non-ST-segment elevation myocardial infarction [13], while ST-segment elevation myocardial infarction is one of the essential causes of acute decompensated heart failure, with a mortality rate of 5% to 8% during hospitalization and a high readmission rate [14]. Recent studies have identified that the majority of patients with ST-segment elevation myocardial infarction have underlying diseases, with diabetes being a common underlying condition [15]. Patients with ST-segment elevation myocardial infarction combined with diabetes have been reported to be on average older and have a higher component of Killip′s cardiac function class ≥ III on admission, with the occurrence of hypertension, hyperlipidemia, three-vessel disease, and left with primary disease. The rate is greater, as is the mortality during hospitalization which was also higher [16].

Glucose management is the primary goal of patients with diabetes [17]. Not only does poor blood glucose control increase the risk of retinal, kidney, and microvascular lesions in diabetic patients [18], but in patients with acute myocardial infarction, adverse fluctuations in blood glucose could exacerbate coronary artery injury [19]. In this study, diabetic patients with myocardial infarction were divided equally into three groups according to their HbA1c levels. The results revealed that patients with HbA1c > 8.5% and 6.5% ≤ HbA1c ≤ 8.5% had significantly higher FBG and HbA1c levels than those with HbA1c < 6.5% and those with HbA1c > 8.5% greater than 6.5% ≤ HbA1c ≤ 8.5%, which is consistent with previous research results [20], indicating that patients with diabetes and myocardial infarction with poor blood glucose control recently have higher FBG, and clinicians should promptly adjust the treatment plan in time to for effective glycaemic control. Glycated haemoglobin is a product of the binding of red blood cell haemoglobin and glucose in the body's blood. When the body's blood glucose is not abnormal, the level of glycated haemoglobin is about 7% of the total haemoglobin and is not affected by age, race, or gender. Haemoglobin glycation is an irreversible process and is a slow, nonenzymatic reaction that correlates with the body's blood glucose concentration and the duration of the presence of high glucose and is not affected by changes in blood glucose [21, 22]. The results of this study suggest that high levels of glycated haemoglobin may be a useful predictor of poor prognosis in patients with acute myocardial infarction combined with diabetes, indicating that poor glycaemic control predisposes to adverse cardiac events. Analysis of the causes may be due to the body's chronic hyperglycaemia, which raises the level of glycated haemoglobin, which in turn reduces the oxygen-carrying capacity of haemoglobin, while chronic hyperglycaemia leads to a reduction in the efficiency of the body's oxygen dissociation, aggravating myocardial hypoxia and ischaemia. High levels of glycated haemoglobin lead to a reduction in the body's ability to compensate for hypoxia, which has an effect on the establishment of collateral circulation and consequently on the recovery of cardiac function. High levels of glycated haemoglobin trigger abnormalities in the body's endothelial function, making the atherosclerotic plaque less stable and increasing the incidence of untoward events [23, 24].

According to the latest ESC guidelines, NT-proBNP has been adopted as a marker for evaluation of heart failure and as an essential indicator of cardiac function and prognosis in patients with acute myocardial infarction [25]. UA is an end product of purine metabolism in vivo, which was previously thought to be associated with renal injury [26]. However, as research has progressed, it has been revealed that UA cannot be applied as an indicator to reflect renal injury but rather as a risk factor for cardiovascular damage [27]. NT-proBNP is an essential risk predictor for cardiovascular disease and is primarily secreted and synthesised by ventricular cells. Clinical studies have found that when patients develop STEMI, structural changes in the heart promote the secretion of synthetic NT-proBNP by ventricular myocytes, which is closely associated with dilatation of the heart chambers, increased ventricular wall tension, and ventricular remodelling in the area of the lesion.

In this study, the levels of NT-proBNP and UA in blood, cardiac color Doppler ultrasound parameters, and NYHA classification were used to evaluate the cardiac function of three groups of patients. And the composition ratio of NYHA grades III and IV was significantly higher than that of HbA1c < 6.5%, and the LVEF was lower than HbA1c < 6.5%, which consistent with the results of previous research [28]. In addition, correlation analysis demonstrated that HbA1c levels were correlated with NT-proBNP, NT-proBNP, UA, LVEDD, LVESD, and NYHA grades which were significantly positively correlated and negatively correlated with LVEF. The above results suggested that HbA1c levels in patients with diabetes combined with myocardial infarction are closely related to the degree of cardiac function damage.

Certain factors may play a key role in the association between HbA1c levels and poor prognosis. Increased HbA1c levels are associated with certain baseline characteristics that elevate the risk of cardiovascular disease, which explains part of the increase in long-term mortality. Additionally, there is a robust association between overt diabetes and adverse cardiovascular outcomes, and it is conceivable that part of the association between poor long-term glycaemic control and outcomes has the same complex mechanisms as the association between overt diabetes and cardiovascular outcomes. Indeed, it is well established that the risk of developing coronary artery disease is not limited to diabetics but exists in other states of impaired fasting glucose, impaired glucose tolerance, and insulin resistance. Reasonable and effective blood glucose control is an important means of reducing cardiovascular complications in patients. In terms of prognosis, the incidence of remyocardial infarction and mortality of patients in group C was significantly higher than those in the groups A and B, further indicating the prognostic importance of glycaemic control on patients' prognosis.

As the proportion of people with chronic poor glycaemic control and consequent cardiovascular disease is likely to increase in the next decade, more appropriate treatment should be recommended for this population. According to the European guidelines for the management of diabetes, prediabetes, and cardiovascular disease, it is recommended that people at high risk of type 2 diabetes should undergo lifestyle modifications. If necessary, medication should be administered to reduce their risk of developing overt hyperglycaemia and type 2 diabetes and, in particular, to prevent or slow down the onset of cardiovascular disease. While this approach has yet to be proven for slowing the course of diabetes, in patients with diabetes or mildly abnormal blood glucose levels, the overall increased risk of cardiovascular disease cannot be explained by abnormalities in blood glucose or HbA1c alone. However, considering that lowering HbA1c levels may have an improved prognosis, it is still possible to encourage our patients to make lifestyle modifications or take medication to prevent or slow down the onset of cardiovascular disease. There are still some limitations to our study. Firstly, this study was conducted in a single centre and is subject to a large margin of error and chance due to the small sample size, limited follow-up time, and small number of cases followed up to the clinical endpoint. Furthermore, as glycated haemoglobin levels were only measured once during hospitalization, it was not feasible to assess the change in HbA1c levels after active treatment and its correlation with clinical events.

## 5. Conclusion

To sum up, the HbA1c levels in diabetic patients combined with myocardial infarction are closely related to the degree of cardiac impairment, and reasonable and effective glycaemic control is of great significance to the prognosis of patients. Considering the possible role of lowering HbA1c levels in improving the prognosis of STEMI, patients with elevated HbA1c should be advised to make lifestyle modifications or take medication to prevent or slow down adverse cardiovascular events. This requires the consideration of clinicians.

## Figures and Tables

**Table 1:** Comparison of general data among the three groups (*n* = 31).

	Group A	Group B	Group C	*F*/*χ*^2^	*P*
Age (year)	68.36 ± 5.12	68.48 ± 5.15	68.54 ± 5.11	0.010	0.990
BMI (kg/m^2^)	22.45 ± 1.63	21.69 ± 1.57	22.23 ± 1.59	1.859	0.1617
Diabetes course (year)	4.21 ± 1.25	4.34 ± 1.23	4.46 ± 1.27	0.310	0.734
Smoking history				0.282	0.869
Yes	20	19	21		
No	11	12	10		
Combined hypertension				0.097	0.953
Yes	21	20	21		
No	10	11	10		
Combined hyperlipidemia				0.602	0.740
Yes	14	16	17		
No	17	15	14		
History of cardiovascular disease				0.313	0.855
Yes	8	9	10		
No	23	22	21		
Hypoglycaemic treatment				1.118	0.572
Oral hypoglycaemic drugs	14	15	18		
Subcutaneous insulin injection	17	16	13		
Infarct site				1.681	0.739
Extensive anterior	15	17	16		
Anterior	8	10	9		
Inferior	8	4	6		

**Table 2:** Comparison of blood glucose indexes among three groups ($\bar{x}\pm s$).

Groups	*n*	FBG (mmol/L)	HbA1c (%)
Group A	31	6.11 ± 0.85	5.46 ± 0.47
Group B	31	7.65 ± 0.94^a^	7.63 ± 0.54^a^
Group C	31	8.94 ± 0.98^ab^	9.88 ± 0.61^ab^
*F*		72.742	513.474
*P*		0.001	0.001

Note: compared with group A, ^a^*P*<0.05; compared with group B, ^b^*P*<0.05.

**Table 3:** Comparison of cardiac function among the three groups (*n* = 31, $\bar{x}\pm s$).

Index	Group A	Group B	Group C	*F*/*χ*^2^	*P*
NT-proBNP (pg/mL)	312.98 ± 63.29	568.36 ± 87.47^a^	918.83 ± 301.48^ab^	83.904	0.001
UA (*μ*mol/L)	308.85 ± 25.46	364.26 ± 29.72^a^	476.83 ± 32.57^ab^	263.155	0.001
LVEDD (mm)	45.28 ± 1.96	49.52 ± 2.07^a^	53.35 ± 2.13^ab^	119.673	0.001
LVESV (mL)	23.12 ± 1.29	28.98 ± 1.35^a^	35.86 ± 1.44^ab^	680.140	0.001
LVEF (%)	49.34 ± 3.31	46.63 ± 3.36^a^	39.11 ± 3.28^ab^	79.156	0.001
NYHA grade				25.385	0.001
I	12/38.71	2/6.45	0/0.00^a^		
II	9/29.03	10/32.26	6/19.35		
III	4/12.90	9/29.03^a^	10/32.26^a^		
IV	6/19.35	10/32.26^a^	15/48.39^ab^		

Note: compared with group A, ^a^*P*<0.05; compared with group B, ^b^*P*<0.05.

**Table 4:** Correlation analysis between HbA1c and various indicators.

Index	HbA1c	
	*r*	*P*
FBG	0.685	0.001
NT-proBNP	0.954	0.001
UA	0.698	0.001
LVEDD	0.962	0.001
LVESD	0.641	0.001
LVEF	-0.867	0.001
NYHA grade	0.713	0.001

**Table 5:** Comparison of prognosis among the three groups *n* (%).

Groups	*n*	Remyocardial infarction (MI)	Death
Group A	31	3/9.68	1/3.23
Group B	31	4/12.90	3/9.68
Group C	31	10/32.26^ab^	8/25.81^ab^
*χ* ^2^		6.190	7.463
*P*		0.045	0.024

Note: compared with group A, ^a^*P*<0.05; compared with group B, ^b^*P*<0.05.

## Data Availability

All data generated or analysed during this study are included in this published article.
